The article "Machine learning approaches for predicting Cracking Tolerance Index (CTIndex) of asphalt concrete containing reclaimed asphalt pavement" was published in 2023. Journal: PLoS One.

# Machine learning approaches for predicting Cracking Tolerance Index (CTIndex) of asphalt concrete containing reclaimed asphalt pavement

**DOI:** 10.1371/journal.pone.0287255

**Published:** 2023-10-26

**Authors:** Lan Ngoc Nguyen, Thanh-Hai Le, Linh Quy Nguyen, Van Quan Tran

**Affiliations:** 1 University of Transport and Communications, Hanoi, Vietnam; 2 University of Transport Technology, Hanoi, Vietnam; Mirpur University of Science and Technology, PAKISTAN

## Abstract

One of the various sorts of damage to asphalt concrete is cracking. Repeated loads, the deterioration or aging of material combinations, or structural factors can contribute to the development of cracks. Asphalt concrete’s crack resistance is represented by the CT index. 107 CT Index data samples from the University of Transport Technology’s lab are measured. These data samples are used to establish a database from which a Machine Learning (ML) model for predicting the CT Index of asphalt concrete can be built. For creating the highest performing machine learning model, three well-known machine learning methods are introduced: Random Forest (RF), K-Nearest Neighbors (KNN), and Multivariable Adaptive Regression Spines (MARS). Monte Carlo simulation is used to verify the accuracy of the ML model, which includes the Root Mean Square Error (RMSE), Mean Absolute Error (MAE), Mean Absolute Percentage Error (MAPE), and coefficient of determination (R2). The RF model is the most effective ML model, according to analysis and evaluation of performance indicators. By SHAPley Additive exPlanations based on RF model, the input Aggregate content passing 4.75 mm sieve (AP4.75) has a significant effect on the variation of CT Index value. In following, the descending order is Reclaimed Asphalt Pavement content (RAP) > Bitumen content (BC) > Flash point (FP) > Softening point > Rejuvenator content (RC) > Aggregate content passing 0.075mm sieve (AP0.075) > Penetration at 25°C (P). The results study contributes to selecting a suitable AI approach to quickly and accurately determine the CT Index of asphalt concrete mixtures.

## 1. Introduction

Asphalt concrete is one of the most common types of pavement surface materials used in the world. Asphalt concrete mixtures are materials with many advantages, such as being easy to construct with high productivity, open to traffic immediately after construction, good quality, uniform, and easy to repair. However, asphalt concrete mixtures are a typically temperature and humidity sensitive material, so in the operation process, under the effect of heavy loads, large vehicle traffic combined with environmental impacts such as high temperatures and humidity, asphalt pavement is easily degraded in quality leading to damage, rutting, permanent deformation, cracking. Cracking is one of many types of damage to asphalt concrete. Cracks develop due to repeated loading, deterioration or aging of material mixtures or structural conditions. All these factors affect the durability of the pavement. Cracks are not early treated, it will widen and grow. Rainwater will penetrate the crack, causing further cracking and possibly leading to structural damage.

The article "Machine learning approaches for predicting Cracking Tolerance Index (CTIndex) of asphalt concrete containing reclaimed asphalt pavement" was published in 2023. Journal: PLoS One.

An extensive literature review conducted as part of the National Cooperative Highway Research Program (NCHRP) 9–57 identified various crack tests [1]. Seven cracking tests were finally selected by the NCHRP 9–57 members and invited experts for further field validation, namely bending beam fatigue (BBF) test, overlay test (OT), disk-shaped compact tension (DCT) test, indirect tensile creep and strength test (IDT-CST) with full instrumentation, and three versions of semi-circular bend (SCB) tests [2]. The above tests have disadvantages such as: cutting samples, long testing time, high cost of equipment, etc.

In 2017, Zhou et al. [2] researched and developed a new test for cracking of asphalt concrete mixture called IDEAL-CT (indirect tensile asphalt cracking test) for determining the CT index representing the crack resistance of asphalt concrete. The IDEAL-CT test is sensitive to the composition of the asphalt concrete mixture and has been carried out at the State Departments of Transportation and in the contractors’ laboratories in the United States. Compared with the above seven concrete cracking test methods, the IDEAL-CT method can be easily implemented with the following advantages: no instrumentation, cutting, gluing, drilling, or notching of specimens) and practicality (minimum training needed for routine operation), and repeatability (coefficient of variance less than 25%) [3, 4]. It is also reported that the CT Index measured in the IDEAL-CT test correlated well with the field performance in terms of fatigue cracking from the FHWA accelerated loading facility full-scale testing.

Yan et al. [5] studied and compared the cracking tolerance index of asphalt concrete mixtures between 3 test methods SCB-IFIT, un-notched SCB-IFIT, and IDEAL-CT. The cracking tolerance index (CT index) results from IDEAL-CT correlate very well with the FI from SCB-IFIT. CT index results show less variation than the FI results (average COV of 5.3% versus 23.0%). Since the IDEAL-CT requires no specimen cutting or notching, it could be a promising alternative to evaluate the cracking resistance of asphalt mixtures.

Standard Test Method for Determination of Cracking Tolerance Index of Asphalt Mixture Using the Indirect Tensile Cracking Test at Intermediate Temperature ASTM D8225-19 has been promulgated by ASTM in 2019. Experimental tests can evaluate the material properties and physical and mechanical properties of the asphalt mixture. However, the time to carry out these tests is quite long and does not provide nearly complete information about the main and essential factors among the variables. Accidentally, in the process of making an error at a certain step, the experiment will have to be repeated, which causes a great loss in cost and time. Therefore, it is necessary to use new approaches to overcome such obstacles.

The article "Machine learning approaches for predicting Cracking Tolerance Index (CTIndex) of asphalt concrete containing reclaimed asphalt pavement" was published in 2023. Journal: PLoS One.

In the past few years, artificial intelligence or Machine Learning (ML) model has been one of the advanced techniques in the industrial 4.0 era that has been applied in many fields of technical science and natural science to solve real-life problems, initially showing outstanding effectiveness and benefits. These methods also predict many essential pavement parameters in the transport sector. Le et al. [6] developed an alternative numerical tool using an artificial neural network (ANN) to predict SMA mixtures’ Marshall Stability and Marshall Flow. Nguyen et al. [7] used an adaptive open neural inference system to predict the international roughness index IRI. Le et al. [8] developed three AI models, namely GAANFIS, PSOANFIS, and Support Vector Machine (SVM), to predict the Marshall Parameters of Stone Matrix Asphalt. The ability and effectiveness of artificial intelligence techniques or ML model in predicting asphalt concrete problems have also been evaluated and confirmed in many other studies [9–11]. Using a classification and regression tree (CART), Arifuzzaman et al. [12] examined the aging behavior of asphalts treated with styrene-butadiene-styrene (SBS) and styrene-butadiene (SB), and carbon nanotube (CNT). Additional explanatory connections between numerous factors that affect how oxidized asphalt behaves at different levels of the tree are revealed by the CART analysis. And it was shown to be more accurate than the outcomes of the regression model. The above studies show that it is feasible to apply artificial intelligence techniques to predict the CT index of asphalt concrete mixtures. Liu et al. [13] used ANN and SVM combining dimensionality reduction techniques as Principal Component Analysis (PCA) for predicting alligator cracking and longitudinal cracking of asphalt pavement. Five different ML algorithms including SVM, RF, ANN and Gradient Boosting (GB), and multiple linear regression were proposed to predict rutting depth of asphalt pavement [14]. In the investigation of Liu et al. [15], international roughness index (IRI) of asphalt pavement is also successfully predicted by machine learning models including SVR, ANN, GB, RF, Gaussian process regression and Extra-trees.

The article "Machine learning approaches for predicting Cracking Tolerance Index (CTIndex) of asphalt concrete containing reclaimed asphalt pavement" was published in 2023. Journal: PLoS One.

In this study, 107 data samples of CT_Index_ were used, each CT_Index_ data sample was determined as the average of three individual samples in the laboratory. The experimental procedure is described in the section 3. Based on these data samples, a database is created to build Machine Learning model to predict CT index of asphalt concrete. Three popular Machine Learning algorithms such ash Random Forest (RF), K-Nearest Neighbors (KNN), and Multivariable Adaptive Regression Spines (MARS) are introduced for building the best performance ML model. The performance of the ML models was assessed using four performance indexes such as the Root Mean Square Error (RMSE), Mean Absolute Error (MAE), Mean Absolute Percentage Error (MAPE), and coefficient of determination (R^2^). The performance of ML model is validated by Monte Carlo simulation. Based on the best performance ML model, SHAPley Additive exPlanations (SHAP value) [16] is a visualization tool that is introduced to make machine learning model’s output more understandable. Therefore, in order to make clear the effect of each input variable including 8 factors such as (1) Aggregate content passing 4.75 mm sieve (AP4.75), (2) Aggregate content passing 0.075 mm sieve (AP0.075), (3) Bitumen content (BC), (4) Penetration at 25°C (P), (5) Flash point (FP), (6) Softening point (°C), (7) Reclaimed Asphalt Pavement content (RAP) and (8) Rejuvenator content (RC) on the CT_Index_, the feature importance analysis will be performed by SHAPley Additive exPlanations in the last section. The study’s results contribute to selecting a suitable AI approach to quickly and accurately determine the CT index of asphalt concrete mixtures.

## 2. Significance research

CT index is a relatively new index introduced to determine the shear resistance of asphalt pavement. However, the experiment to determine CT index of asphalt pavement is relatively expensive and time consuming. Application of machine learning models has been carried out to study many properties of pavement. However, the study of CT index by machine learning model has not been proposed. Therefore, this study focuses on proposing to build a high performance machine learning model to evaluate CT index from 8 input boundaries including (1) Aggregate content passing 4.75 mm sieve (AP4.75), (2) Aggregate content passing 0.075 mm sieve (AP0.075), (3) Bitumen content (BC), (4) Penetration at 25°C (P), (5) Flash point (FP), (6) Softening point (°C), (7) Reclaimed Asphalt Pavement content (RAP) and (8) Rejuvenator content (RC), and evaluate and quantify the influence of these input variables on the CT index value.

The article "Machine learning approaches for predicting Cracking Tolerance Index (CTIndex) of asphalt concrete containing reclaimed asphalt pavement" was published in 2023. Journal: PLoS One.

## 3. Experimental procedure and experimental results

### 3.1. Material used

The asphalt mixtures used in the evaluation are shown in Table 1 with Dense Graded Asphalt (DGA) and gab-grade of Stone Matrix Asphalt (SMA). The two sources of aggregate used for the mixtures are designated type I and type II, respectively. The properties of these two aggregate sources are shown in Table 2.

**Table 1:** Labels of various mixtures in database.

Mixture type	Code	RAP content	Asphalt type	Rejuvenator	Aggregate source^(^^*^^)^
DGA	B1	0%	PMB III	-	I
DGA	B2	0%	PMB III	1.5% Sasobit	I
SMA	B1	0%	PMB III	-	I
SMA	B2	0%	PMB III	1.5% Sasobit	I
DGA	B3	0%	60/70	1.5% Sasobit	II
DGA	B3	20%	60/70	1.5% Sasobit	II
DGA	B3	30%	60/70	1.5% Sasobit	II
DGA	B3	40%	60/70	1.5% Sasobit	II
DGA	B3	50%	60/70	1.5% Sasobit	II
DGA	B4	0%	60/70	0.15% Zycotherm	II
DGA	B4	20%	60/70	0.15% Zycotherm	II
DGA	B4	30%	60/70	0.15% Zycotherm	II
DGA	B4	40%	60/70	0.15% Zycotherm	II
DGA	B4	50%	60/70	0.15% Zycotherm	II
DGA	B5	30%	60/70	3.0% Prephalt	II
DGA	B6	40%	60/70	5.0% Prephalt	II
DGA	B7	50%	60/70	7.0% Prephalt	II

^(*)^aggregate source: Type I: Khau Dem, Lang Son, Vietnam, Type II: Tan Cang, Bien Hoa, Dong Nai, Vietnam.

**Table 2:** Aggregate properties.

Properties	Agg.19		Agg.12.5		Agg.9.5		Agg.4.75	
	I	II	I	II	I	II	I	II
Bulk Specific Gravity (g/cm^3^)	2.865	2.724	2.847	2.734	2.824	2.726	2.794	2.702
Apparent Specific Gravity (g/cm^3^)	2.923	2.773	2.918	2.753	2.876	2.753	2.894	2.740
Water absorption, %	0.697	0.65	0.846	0.204	0.741	0.366	1.248	0.517
Los Angeles abrasion, %	9.4	16.25	11.8	20.5	10.53	15.32	-	-
Flat and elongation, %	8.7	6.88	10.4	11.1	7.82	11.25	-	-
Clay, dust content, %	0.5	0.62	0.9	0.31	0.47	0.76	1.8	1.7
Sand Equivalent-SE, %	-	-	-	-	-	-	88.1	74.6
Fine Aggregate Angularity, %	-	-	-	-	-	-	51.7	49.3

According to AASHTO M323, Agg.19: Nominal Maximum Aggregate Size of 19 mm; Agg.12.5: Nominal Maximum Aggregate Size of 12.5 mm; Agg.9.5: Nominal Maximum Aggregate Size of 9.5 mm; Agg.4.75: Nominal Maximum Aggregate Size of 4.75 mm.

Valdés et al. [17] shows the acceptable range of Reclaimed Asphalt Pavement (RAP) varying from 10% to 50% weight of asphalt pavement. Three types of rejuvenator consisting of sasobit, Zycotherm and Prephalt are used as additive binder for Dense Graded Asphalt (DGA) According to Anderson et al. [18], the sasobit content as 1.5% weight of binder should be used. Ayazi et al. [19] proposed the used Zycotherm to be equal to 0.15% weight of binder. Three contents of prephalt including 3.0, 5.0 and 7.0% weight of binder are recommended to use according to Shi et al. [20]. Therefore, the study also used cracking test data of Warm Mixtures Asphalt (WMA) and Hot Mixtures Asphalt (HMA) with RAP content of 0%, 20%, 30%, 40% and 50% weight of binder, respectively, to analyze accumulate. The WMA uses Sasobit and Zycotherm additives, HMA uses Prephalt rejuvenator additive at the contents of 3%, 5% and 7% respectively. The properties of the virgin and modified binders in unaged condition are shown in Table 3.

The article "Machine learning approaches for predicting Cracking Tolerance Index (CTIndex) of asphalt concrete containing reclaimed asphalt pavement" was published in 2023. Journal: PLoS One.

**Table 3:** Properties of asphalt binders.

	Virgin binder (Bitumen 60/70)	B1 (Bitumen PMB III)	B2 (Bitumen PMB III with 1.5% Sasobit)	B3 (Bitumen 60/70 with 1.5% Sasobit)	B4 (Bitumen 60/70 with 0.15% Zycotherm)	B5 (Bitumen 60/70 with 3.0% Prephalt)	B6 (Bitumen 60/70 with 5.0% Prephalt)	B7 (Bitumen 60/70 with 7.0% Prephalt)
Penetration at 25°C	64	52	42	52	64	61	63	66
Flash point,°C	254	249	271	247	259	248	242	237
Softening point,°C	49.6	88	94	69.8	50.7	54	51.4	49.3
Ductility at 25°C, cm	>100	>100	>100	>100	>100	>100	>100	>100

Flash point should have the significant effect on performance of asphalt pavement at high temperature, and Penetration at 25°C seems to have not any meaningful of binder performance. In this study, the results of CT index testing of asphalt mixes using 5 types of bitumen binder are described in Table 1. To distinguish 5 types of bitumen binder for the CT index evaluation test in unaged condition, four properties including Flash point, Penetration at 25°C, Softening point and Ductility at 25°C described in Table 3 are considered, properties of bitumen binder for Short-term aged (RTFO) and Long-term aged (PAV) are not considered in this investigation. Ductility at 25°C of the 5-bitumen binders has similarity value (> 100 cm). Evaluating the influence of bitumen binders’ properties on CT index by ML technique-SHAP value is also the aim of this study.

Therefore, 3 input variables including Flash point, Penetration at 25°C and Softening point are used to build a machine learning model to determine and evaluate the CT index.

The study used asphalt mixtures currently used in Vietnam, these mixtures were designed according to the Marshall method. When preparing the CT_index_ test sample, the gyratory compaction is used to ensure the air voids of the mixture according to the regulations of ASTM D8225 is equal to be 7±0.5%. There are 17 mixtures of DGA and SMA designed according to Marshall method, the specifications of the mixtures all meet the specifications according to MS-02 and AASHTO M325. Fig 1 shows the gradation curves of a mixture of SMA and DGA designed using aggregate type I and II.

**Fig 1:** Mixture gradation aggregates: (a) Stone Mastic Asphalt (SMA) samples, (b) Dense Graded Asphalt (DGA) samples.

The article "Machine learning approaches for predicting Cracking Tolerance Index (CTIndex) of asphalt concrete containing reclaimed asphalt pavement" was published in 2023. Journal: PLoS One.

### 3.2 Methodology of experiment

The IDEAL-CT was used to determine the intermediate-temperature cracking resistance of asphalt mixtures. The indirect tensile asphalt cracking test was recently developed as a practical cracking test that could be routinely used in asphalt mix design as well as for quality control/quality assurance (QC/QA) [2]. The test is performed on 150-mm diameter and 62-mm high gyratory specimens that are typically compacted to a target air void level of 7 ± 0.5 percent. Test specimens are conditioned for two hours at 25°C, and then tested using an indirect tension load frame. A minimum of three replicates are typically tested for a mixture. Testing can be performed using a stand-alone servo-hydraulic machine capable of sampling load and displacement data at a rapid rate (40 Hz), as shown in Fig 2(A). Specimens are loaded monotonically at a rate of 50 mm/min in load line displacement (LLD) until failure. A plot of load versus LLD is shown in Fig 2(B). The plot of load versus displacement is then analyzed to determine the CT index:

$${\text{CT}}_{\text{index}}=\frac{\text{t}}{\text{62}}\times \frac{{\text{G}}_{\text{f}}}{\left|{\text{m}}_{\text{75}}\right|}\times \left(\frac{{\text{l}}_{\text{75}}}{\text{D}}\right)$$ (1)

where:

G_f_−fracture energy, J/m^2^

|m_75_| ‐ slope at 75% peak load, N/m

D ‐ specimen diameter, mm

t ‐ specimen thickness, mm

l_75_ ‐ displacement corresponding to 75% of the peak load at the post-peak stage, mm

**Fig 2:** IDEAL-CT Test Device and Typical Result: (a) Test Device; (b) Recorded Load (P) versus Load-Line Displacement Curve according to Zhou et al [2].

The specimen diameter D is the standard value 150 mm; therefore, this is a constant which can be neglected. Moreover, the Eq (1) helps to calculate experimentally CT index value in the experimental part (2.1 and 2.2 of this study). Therefore, the specimen diameter D is not considered in for building Machine Learning model in the next sections.

### 3.3. Experimental results and analysis

In this study, the database on cracking tolerance index CT_Index_ was collected from experimental studies in the laboratory of the University of Transport Technology. The database includes 107 records on the CT_Index_ cracking tolerance index of asphalt mixtures, SMA mixes, and Reclaimed asphalt pavement (RAP) using common asphalt, polymers, and additives, such as Sasobit, Zycotherm, and Prephalt.

The input data includes 8 variables: (1) Aggregate content passing 4.75 mm sieve (AP_4.75_), (2) Aggregate content passing 0.075 mm sieve (AP_0.075_), (3) Bitumen content (BC), (4) Penetration at 25°C (P), (5) Flash point (FP), (6) Softening point (°C), (7) Reclaimed Asphalt Pavement content (RAP) and (8) Rejuvenator content (RC) on the CT_Index_. The output data is the cracking tolerance index CT_Index_ (CT).

The article "Machine learning approaches for predicting Cracking Tolerance Index (CTIndex) of asphalt concrete containing reclaimed asphalt pavement" was published in 2023. Journal: PLoS One.

The dataset used in the study was randomly divided into two sub-datasets using a uniform distribution, in which 70% of the data was used to build the training model and 30% of the data was used for verification. The statistical parameters such as minimum, median, maximum and standard deviations… are presented in detail in Table 4.

**Table 4:** Description of database used in this study.

	Sym	Count	Mean	Std	Min	Q_25%_	Median	Q_75%_	Max	Skw
Aggregate content passing 4.75 mm sieve (%)	AP_4.75_	107	46.93	7.09	24.80	45.20	49.50	50.70	53.10	-2.29
Aggregate content passing 0.075 mm sieve (%)	AP_0.075_	107	8.02	1.03	6.40	7.10	8.40	8.80	9.60	-0.09
Bitumen content (%)	BC	107	4.91	0.76	3.50	4.55	5.10	5.20	6.70	0.20
Penetration at 25°C (mm)	P	107	59.49	7.31	43.00	52.00	64.00	64.60	66.00	-0.98
Flash point (°C)	FP	107	290.54	48.39	247.00	248.00	259.00	351.00	362.00	0.54
Softening Point	SP	107	59.38	15.94	48.00	48.20	50.70	69.80	95.00	1.22
Reclaimed Asphalt Pavement content (%)	RAP	107	22.43	19.32	0.00	0.00	30.00	40.00	50.00	0.01
Rejuvenator content (%)	RC	107	1.26	2.33	0.00	0.00	0.00	1.50	7.00	1.56
CT_Index_	CT	107	138.89	136.96	16.89	62.50	97.31	158.61	638.67	2.61

Sk = Skewness; Std = Standard deviation

Fig 3 depicts the distribution of input parameters in this study. The plots for the distribution of the data for the parameters are shown through the histograms from Fig 3A–3H. Most of the variation in the number of samples has a relatively large distribution, often concentrated in a relatively narrow range of values. Aggregate content passing 4.75 mm sieve (AP4.75) varied from 24.8% to 53.1%, with most samples in the 50% content range. Aggregate content passing 0.075 mm sieve (AP0.075) ranges in content from 6.4% to 9.6%. A fairly large number of samples are concentrated in the 7% range, others in the 8–9% range. Bitumen content (BC) has a large number of samples in the 5% range. Penetration at 25°C (P) has the number of samples located mainly in the range of 60–65 g/cm^3^. Flash point (FP) ranges from 247-362(mm), but most data points are in the 250–275 mm range. Softening point has distribution values concentrated mainly at 50°C. With Reclaimed Asphalt Pavement content (RAP) and rejuvenator content (RC) visible, most samples are concentrated in the 0% range. The distribution of the number of samples of the output variables in the experimental data (Fig 3I) shows that most of the samples have the CT index value of cracking tolerance index in the range of 0–200.

**Fig 3:** Distribution of input variable (a) Aggregate content passing 4.75 mm sieve (AP4.75), (b) Aggregate content passing 0.075 mm sieve (AP0.075), (c) Bitumen content (BC), (d) Penetration at 25°C (P), (e) Flash point (FP), (f) Softening point, (g) Reclaimed Asphalt Pavement content (RAP), (h) Rejuvenator content (RC), and (i) CT Index.

The article "Machine learning approaches for predicting Cracking Tolerance Index (CTIndex) of asphalt concrete containing reclaimed asphalt pavement" was published in 2023. Journal: PLoS One.

The correlation matrix of the input experimental data is depicted in Fig 4. As can be seen, most of the parameters have an influence on the output CT index. The highest observed correlation coefficient between input and output variables is -0.87. In addition, the input parameters also have a significant correlation with each other, expressed through the correlation coefficients between them, with the highest coefficient equal to -0.96. Therefore, the relationships between these variables need to be analyzed further.

**Fig 4:** Pearson correlation between inputs variables and CTindex.

In actuality, the quantity, quality, and number of features (number of input variables) are the key determinants of a machine learning model’s accuracy. The quantity of data and number of characteristics might vary depending on each situation, such as a medical, pharmacological, or civil engineering challenge. For instance, there are a ton of Machine Learning research into the mechanical characteristics of concrete, such as compressive strength, elastic modulus, shear strength, and tensile strength, as well as the properties of soil, such as UCS, CBR, resilient modulus, and coefficient of permeability. Jeremiah et al. [21] identified 23 Machine Learning experiments for soil parameters, with data ranging from 49 to 283 samples and features from 4 to 14. Chaabene et al. [22] compiled the results of 47 Machine Learning experiments on the mechanical characteristics of concrete. In the 47 investigations, there are between 74 and 2817 samples of data, and there are between 4 and 13 characteristics. The computing time is significantly influenced by the number of characteristics. The accuracy and performance of a machine learning model with the same quantity of data and features heavily depend on the machine learning method. As a result, even when there are limited data and numerous features, choosing the right Machine Learning method can assist to increase the model’s capacity for prediction.

The authors of this paper use 3 machine learning algorithms, Random Forest (RF), K-Nearest Neighbors (KNN), and Multivariate Adaptive Regression Splines (MARS), with 107 data points and 8 features to investigate the choice of the best machine learning model. In addition, 8 characteristics are required to study how each input affects the CT index using Shapley Additive Explanation based on ML models. Monte Carlo simulation has been used to confirm the ML model’s dependability. The min-max value range of the variable indicated in Table 4 of the revised paper should be the only range in which the Machine Learning model of this study is used.

The article "Machine learning approaches for predicting Cracking Tolerance Index (CTIndex) of asphalt concrete containing reclaimed asphalt pavement" was published in 2023. Journal: PLoS One.

## 4. Machine learning methods

### 4.1 Random forest (RF)

Fig 5 presents briefly the process of Random Forest algorithm according to conception of Breiman [23]. The random forest (RF) algorithm is a supervised ML algorithm [23]. As the name, it is used to somehow create a forest and make it random. The number of trees in the forest is directly related to the results obtained by the algorithm: the more trees, the more accurate the output. But it should be highlighted that creating a forest is not equivalent to using information gain or creating an index to make a decision. It uses a tree-like graph to show possible results. If a training set with targets and features is input into a decision tree, it will show some regularities. These regularities can then be utilized to make predictions. The process of collecting these information nodes and forming rules is the process of using the information gain method and Gini coefficient calculation. To obtain an objective estimate of the test set error in RF, neither cross-validation nor a separate test set is required. Internally, it is computed using extrapolation from the categorization of the excluded person. Numerous studies have shown that the out-of-bag estimate is unbiased [24, 25]. The difference between the random forest algorithm and the decision tree algorithm is that in the random forest, the process of finding the root node and dividing the characteristic nodes will be carried out in a random manner.

**Fig 5:** Process of Random Forest algorithm according to conception of Breiman [23].

### 4.2 K-Nearest Neighbors (KNN)

K-Nearest Neighbors (KNN) is a common classification and regression algorithm. Determine the kind of the object by looking at its neighbors. Based on the similarity in a covariate space between the population unit for which a prediction is intended and the sample units for which data are provided, the KNN technique and its modifications are intuitive, non-parametric approaches to either univariate or multivariate prediction [26, 27]. Usually, the distance between an object and its neighbors uses the Euclidean distance. In j-dimensional space Euclidean distance of points a(*x*_*1*_, *x*_*12*_, …, *x*_*1j*_) and b(*x*_*2*_, *x*_*22*_, …, *x*_*2j*_) and N objects closest to the object to be checked

$$d_{ab}=\sqrt{\sum_{j=1}^{N}\left(x_{1j}-x_{2j}\right)}$$ (2)

A large collection of training data or objects of the known kind is required for KNN. The premise is that if the nearest item is “a”, then the unknown thing must be “a”, but if the next j nearest objects all is “b”, then the unknown object must be “b”. Normally, no simple voting mechanism is used; each neighbor’s vote is weighted depending on its distance from the unknown object, so closer objects have a greater voice in recognizing it. The disadvantage of the k-neighbor algorithm is that it cannot give any basic structure information about the data, so cannot know what characteristics the average instance sample and the typical instance sample have.

The article "Machine learning approaches for predicting Cracking Tolerance Index (CTIndex) of asphalt concrete containing reclaimed asphalt pavement" was published in 2023. Journal: PLoS One.

### 4.3 Multivariate Adaptive Regression Splines (MARS)

Multiple Adaptive Regression Splines (MARS) is a form of regression analysis introduced by Friedman [28], which is a non-parametric regression technique that can be seen as an extension of a linear model that simulates the nonlinearity and interaction between variables, a general insertion points for the MARS model. It is a nonlinear, nonparametric regression method based on a segmentation strategy. This method does not need to assume a potential specific functional relationship between the input variable and the output variable but divides the data training set into independent sections, line segments, with different gradients, and each segment is called a basis function; the endpoint of each segment is nodes, a node marks the end of one region of data and the beginning of the next. The resulting basis functions will give the model greater flexibility, allowing bending and threshold values that deviate from linearity. MARS generates basis functions through a stepwise search and uses an adaptive regression algorithm to select node locations. The MARS algorithm is divided into two steps: forward selection and backward pruning: the forward selection process is to divide the input sample data, use the spline function instead of the divided cells to fit to get a new basis function, and then get a fitting model; the backward pruning process is to screen the generated basis functions, and eliminate the basis functions that contribute less to the model fitting, so as to avoid overfitting and generate the optimal model. MARS is a data modeling process. Due to make the model conform to the formula, the forward selection procedure should be performed on the training set of the data to make the model conform to the formula. The training error is reduced as much as possible by using the constant term and basis function pair to generate the model; for a model containing N basis functions, the next pair of basis functions added to the model is obtained by the least square method. When a new basis function is added to the model, its interaction with the existing basis functions in the model is also considered. If the number of basis functions reaches the maximum number predetermined by the model, an overfitting model will be generated. The numerator is the mean square error of the MARS model data training set, and the denominator is the penalty function. The more the model complexity, the greater the variance.

The article "Machine learning approaches for predicting Cracking Tolerance Index (CTIndex) of asphalt concrete containing reclaimed asphalt pavement" was published in 2023. Journal: PLoS One.

### 4.4 Performance evaluation of models

Model assessment is a crucial step in the development of a machine learning model that determines if the model is of high quality.

In order to use the proper assessment measures, model evaluation aids in the selection of models that are appropriate for a given situation. The coefficient of determination (R^2^), the root mean square error (RMSE), the mean absolute error (MAE), and the mean absolute percent error (MAPE) were the four statistical performance metrics employed in this investigation [25].

The following criteria establish these ratings:

$$R^{2}=1-\left[\frac{\Sigma_{j=1}^{N}{\left(M_{j}-Q_{j}\right)}^{2}}{\Sigma_{j=1}^{N}{\left(M_{j}\right)}^{2}}\right]$$ (3)

$$RMSE=\sqrt{\frac{1}{N}\overset{N}{\underset{j=1}{\Sigma }}{\left(M_{j}-Q_{j}\right)}^{2}}$$ (4)

$$MAE=\frac{1}{N}\overset{N}{\underset{j=1}{\Sigma }}|M_{j}-Q_{j}|$$ (5)

$$MAPE=100\frac{1}{N}\sum_{j=1}^{N}\frac{\left|M_{j}-Q_{j}\right|}{M_{j}}$$ (6)

Where *M*_*j*_ is the experimental value of CT index, *Q*_*j*_ is the predicted value and N is the number of samples.

### 4.5 Methodology flowchart

The general outline of the predicted cracking tolerance index of asphalt concrete mixtures is detailed in Fig 6. This flowchart consists of three main steps, as follows: Step 1: The data used in this study were collected from the laboratory with the 107 samples presented in Section 2.3 earlier. These data include 8 inputs: Aggregate content passing 4.75 mm sieve (AP4.75), aggregate content passing 0.075 mm sieve (AP0.075), bitumen content (BC), penetration at 25°C(P), flash point (FP), softening point (SP), Reclaimed asphalt pavement content (RAP), and rejuvenator content (RC). The output is the cracking tolerance index CTindex (CT). This data is randomly split into two datasets, with 70% used for training the models and the remaining 30% for testing.

**Fig 6:** Outline of model building.

Step 2: The math facts are trained to perform the CT index prediction task, the model is built, and it is selected with an appropriate structure.

Step 3: Validate the model. Models are tested and validated using test datasets. The predictive ability of the models was evaluated through the criteria R^2^, RMSE, MAE, and MAPE. The model with optimal performance will be selected to predict the CT index and analyze the sensitivity to evaluate the influence of input parameters on the CT index.

The article "Machine learning approaches for predicting Cracking Tolerance Index (CTIndex) of asphalt concrete containing reclaimed asphalt pavement" was published in 2023. Journal: PLoS One.

## 5. Results and discussion

### 5.1 Performance evaluation of predictive machine learning algorithms

Fig 7 shows the accuracy of the training and testing model. Predictive performance is evaluated across four metrics, namely R2, RMSE, MAE, and MAPE. It can be observed that the RF and MARS models have R2 values on the training and testing datasets that are relatively similar (Fig 7A). Which, the RF model has a higher R^2^ value than the other two models with an average R^2^ value on the training set of 0.9927, and 0.9757 on the test data set. In the test data set, RF model can achieve R^2^ max value up to 0.9953. Similarly, looking at Fig 7B–7D, it is easy to see that the KNN model has the poorest performance with the RMSE, MAE, and MAPE indices always achieving much larger values than the two MARS and RF models. Indeed, the average performance of the predictive models is presented in Table 5. The mean value of the RMSE index for the KNN model on the training set is 25.2973 and RMSE = 34.7225 on the test set. This is up to two times larger than RF with RMSE = 11.2123 on the training set and RMSE = 17.4854 on the test set. Besides considering the mean value of the evaluation criteria, the standard deviation of the performance values is also considered to comprehensively compare the predictive performance of the models. The table of standard deviation values of the three models on the two training and test data sets is listed in Table 5. The RF model has a slightly smaller standard deviation score than the other two models with precision The standard deviations of the performance indicators R^2^, MAE, and MAPE are 0.0260, 2.8049, and 0.0294, respectively. This result shows that the RF model has superior accuracy compared to MARS and KNN. In addition, the relatively small deviation avoids causing large differences in the prediction performance of the model.

**Fig 7:** Performance value of machine learning models after 3000 simulations (a)R^2^, (b) RMSE, (c) MAE and (d) MAPE values.

**Table 5:** Comparison of three algorithms for compressive prediction using mean performance value and Std performance value.

		Algorithm	Training dataset				Testing dataset			
			R2	RMSE	MAE	MAPE	R2	RMSE	MAE	MAPE
Mean		KNN	0.6778	17.8333	13.7243	0.1427	0.0205	16.9889	13.7467	0.1316
	Min	MARS	0.8986	13.0875	9.8979	0.1036	0.5267	12.0619	9.1206	0.0951
		**RF**	0.909	8.0145	6.1945	0.0603	0.5827	**8.7536**	**7.2763**	**0.0744**
		KNN	0.9599	25.2973	18.4408	0.1898	0.9168	34.7225	25.8973	0.2591
	Average	MARS	0.9826	17.2728	13.6917	0.1577	0.965	21.4317	16.91	0.1894
		**RF**	**0.9927**	**11.2123**	**8.3328**	**0.0838**	**0.9767**	**17.4854**	**13.3076**	**0.1356**
		KNN	0.9866	46.7155	25.1125	0.2387	0.9812	153.6081	88.6094	0.466
	Max	MARS	0.9922	33.2283	27.6053	0.3583	0.9921	295.3152	100.011	0.6597
		**RF**	0.9971	21.9176	10.5877	0.1032	**0.9953**	86.686	48.7802	0.3402
StD		KNN	0.0311	4.5074	1.6728	0.0143	0.0744	12.7486	6.8638	0.0479
		MARS	0.0093	3.1811	2.4928	0.0316	0.0371	4.2467	3.1694	0.0434
		**RF**	0.0032	0.9774	0.6221	0.0064	**0.026**	**4.6759**	**2.8049**	**0.0294**

The article "Machine learning approaches for predicting Cracking Tolerance Index (CTIndex) of asphalt concrete containing reclaimed asphalt pavement" was published in 2023. Journal: PLoS One.

### 5.2 Prediction of typical machine learning algorithm

After the models’ rankings are validated by performance evaluation, the model that can run consistently and with exceptional performance will be chosen. Fig 8 compares the actual value and the predicted value of the RF model. Observe the difference between the experimental value and the predicted value from the RF model. The predicted values of RF on the training set are quite comparable to the training data as red round points. The prediction results obtained on the test set are surprisingly accurate with the predicted values very close to the true value (blue squares).

**Fig 8:** Comparison between true and predicted CT index of Random Forest model for training and testing set.

It can be observed that the predicted values are very close to the fit line with the evaluation indexes on the experimental data set, which are R^2^ = 0.9953, RMSE = 8.7535, MAE = 7.2763, and MAPE = 0.0795, respectively. The error values between the experimental value and the predicted value for the training data set and the test data are compared in Fig 9. Based on the brown frequency distribution line, the error frequency can easily be seen in samples in the range. For the training database, the frequency of samples with errors in the range [-10;10] is about 5. Similar to the testing set, the frequency of samples with errors in the range [-10;10] is about 3. Finally, it can be concluded that the RF model is capable of predicting CT index of asphalt mixtures with good performance and reliable results.

**Fig 9:** Error value between predicted and true CT index of asphalt concrete (a) training part, (b) testing part.

In Fig 8, eight data samples including 6 data samples for training dataset and 2 data samples for testing dataset have CT index value higher than 200 are identified. These CT index value belong to Stone mastic asphalt (SMA) mixtures using Sasobit and without Sasobit additive. The SMA blend has a high binder content, while using cellulose fibers. The cellulose fibers in the SMA blend have the ability to cross and cross, forming a spatial network structure, this type of structure has the effect of transmitting force while preventing the slip between the particles, the overall connection of the mixture, and the resistance. resist and retard the formation and growth of cracks. Therefore, the SMA composite has better performance than the BTNC blend in terms of top-down crack resistance, bottom-up crack resistance and thermal crack resistance. This conclusion is consistent with the results of Wu et al. [29] and Habbouche et al. [30].

The article "Machine learning approaches for predicting Cracking Tolerance Index (CTIndex) of asphalt concrete containing reclaimed asphalt pavement" was published in 2023. Journal: PLoS One.

In this study, 3 machine learning algorithms including RF, KNN and MARS to build machine learning models for predicting CT index. These machine learning algorithms have hyperparameters which can be (i) tuned for each specific case or (ii) defaults values defined in the open-source library of language programming Python [25]. In this study, the default hyperparameters of three ML algorithms are used. Based on the database including 107 samples and 8 input variables, 3 algorithms are fitted on 70% of the database samples and 8 input variables to predict CT index.

Machine learning models can solve very complex problems, non-linear correlations such as CT index prediction with high accuracy, but the disadvantage of RF, KNN and MARS machine learning models cannot provide equations describing the correlation between outputs and variables as empirical [31]. Therefore, in order to increase the applicability of the RF machine learning model with high performance in predicting CT index and designing pavement components, an excel file derived from the RF model allows predicting CT index by excel formulas (including logic function) attached to this study (S1 File).

### 5.3 Feature importance analysis

The cracks, a common road surface disease, often do not attract people’s attention, and these are only regarded as normal asphalt aging phenomena. However, in recent years, the phenomenon of road surface subsidence caused by road cracks and traffic accidents has occurred from time to time. The cracks like scars are dormant on the road, and with the erosion of rainwater and the increase of vehicle load, they continue to spread vertically and horizontally and may cause collapse at any time [13]. On the other hand, the appearance of cracks will also increase road maintenance’s difficulty and the burden of later road maintenance. Many studies on the influence of composition and manufacturing methods on the mechanical behavior of asphalt mixtures [32–34]. In the study by Sangsefidi et al. [35], two gradations (fine-graded and coarse-graded) were evaluated with two levels of binder content and air voids content to reflect, respectively, construction variable levels of binder content and density. Rutting, tensile cracking, and moisture susceptibility were the three characteristics of mixture performance that were assessed. It has been discovered that for estimating rutting performance, the volume content is more useful than the weight content and that the effective binder content should be considered rather than the overall binder content. Without further breakdown into effective binder content and absorbed binder content, the total binder content may adequately characterize the indirect tensile strength (ITS) values for tensile cracking. Gradation deviation had no discernible impact on cracking.

The article "Machine learning approaches for predicting Cracking Tolerance Index (CTIndex) of asphalt concrete containing reclaimed asphalt pavement" was published in 2023. Journal: PLoS One.

There are 8 data inputs including Aggregate content passing 4.75 mm sieve (AP4.75), Aggregate content passing 0.075 mm sieve (AP0.075), Bitumen content (BC), Penetration at 25°C (P), Flash point (FP), Softening point, Reclaimed Asphalt Pavement content (RAP), and Rejuvenator content (RC). The SHAP values of these data are calculated, and the results are summarized in Fig 10. These data are sorted from top to bottom according to their influence on the CT index output (cf. Fig 10B). With the SHAP values, the picture of feature importance is created clearer, and more abstract, with blue for low values, and gradually red for high values (cf. Fig 10A). Looking at the plot, it is easy to see that SG is the least important feature, and AP4.75 is the feature that has a great influence on the CT index. Based on color, with AP4.75 and RAP feature, with high values (red) SHAP values will be low, so it will push towards layer 0. By SHAPley Additive exPlanations based on RF model, the input Aggregate content passing 4.75 mm sieve (AP4.75) has a significant effect on the variation of CT Index value. In following, the descending order is Reclaimed Asphalt Pavement content (RAP) > Bitumen content (BC) > Flash point (FP) > Softening point > Rejuvenator content (RC) > Aggregate content passing 0.075mm sieve (AP0.075) > Penetration at 25°C (P).

**Fig 10:** SHAP value for feature importance analysis of CT index prediction.

## 6. Conclusions

In this study, RF, KNN, and MARS models are developed to predict the cracking tolerance index of asphalt concrete mixtures. 107 experimental results were collected to build databases and develop models. In which, 70% of the data is randomly selected for the training phase and the remaining 30% is used for the testing phase of the machine learning models. Through analysis and evaluation of performance indicators, the RF model is the most stable and has predictive results close to the real value. On the test set, the RF model has R^2^, RMSE, MAE, and MAPE values of 0.9953, 8.7535, 7.2763, and 0.0795, respectively. Through sensitivity analysis, it can be seen that the crack resistance CT index varies greatly for different combinations of input variables. Of which, Aggregate content passing 4.75 mm sieve (AP4.75) has a significant effect on the variation of CT Index output. Next is Reclaimed Asphalt Pavement content (RAP) > Bitumen content (BC) > Flash point (FP) > Softening point > Rejuvenator content (RC) > Aggregate content passing 0.075 mm sieve (AP0.075) > Penetration at 25°C (P). In addition, the correlation between the input variables is quite complex, which cannot be reflected by a clear equation. The study has quantified the influence of the parameters on the output results, supporting the design of the optimal composition for asphalt concrete in the future. The number of data used in this study is relatively small, which affects the general application of machine learning models in predicting CT index. Therefore, the addition of data samples to the database is very necessary in further studies to build a highly universal machine learning model to improve the applicability of the machine learning model in designing mixture asphalt pavement including SMA using RAP.

The article "Machine learning approaches for predicting Cracking Tolerance Index (CTIndex) of asphalt concrete containing reclaimed asphalt pavement" was published in 2023. Journal: PLoS One.

## Supporting information

S1 File (XLSX)
